# Biogenic Synthesis of Cu-Doped ZnO Photocatalyst for the Removal of Organic Dye

**DOI:** 10.1155/2022/8081494

**Published:** 2022-05-04

**Authors:** Biruktait Ayele Lemecho, Fedlu Kedir Sabir, Dinsefa Mensur Andoshe, Noto Susanto Gultom, Dong-Hau Kuo, Xiaoyun Chen, Endale Mulugeta, Temesgen D. Desissa, Osman Ahmed Zelekew

**Affiliations:** ^1^Department of Materials Science and Engineering, Adama Science and Technology University, Adama, Ethiopia; ^2^Department of Applied Chemistry, Adama Science and Technology University, Adama, Ethiopia; ^3^Department of Materials Science and Engineering, National Taiwan University of Science and Technology, Taipei 10607, Taiwan; ^4^College of Materials Engineering, Fujian Agriculture and Forestry University, Fuzhou 350002, China

## Abstract

The Cu-doped ZnO photocatalysts were prepared with a green and coprecipitation approach by using water hyacinth (*Eichhornia crassipes*) aquatic plant extract. In the preparation process, different amount of copper precursors such as 1, 2, 3, 4, and 5% of molar ratio were added to zinc nitrate precursors and abbreviated as Cu-ZnO (1%), Cu-ZnO (2%), Cu-ZnO (3%), Cu-ZnO (4%), and Cu-ZnO (5%), respectively. The characterization of the obtained samples was carried out, and the removal of the methylene blue (MB) dye was examined. Out of all catalysts, Cu-ZnO (3%) had the best photocatalytic performance and 89% of the MB dye was degraded. However, the degradation performances of blank (without catalysts), ZnO, Cu-ZnO (1%), Cu-ZnO (2%), Cu-ZnO (4%), and Cu-ZnO (5%) catalysts were 6, 54, 69, 83, 80, and 73%, respectively. Therefore, the use of water hyacinth plant extract with the optimum amount of Cu added to ZnO during the preparation of the catalyst could have a promising application in the degradation of organic pollutants.

## 1. Introduction

In recent years, the textile, paper and pulp, and dyeing industries have been developed and put significant pollution into natural water supplies [1–4]. Among the pollutants, organic dyes account for the majority of these contaminants, and they have several negative health effects [5–7]. Therefore, a lot of industrial wastewater treatment methods have been used for the degradation of organic dyes [8, 9]. Among methods, photocatalysis is the best option since it is a green technique that employs naturally renewable solar energy and functioned at room temperature and pressure [10–14]. Recently, semiconductor photocatalysts such as TiO_2_ [15], ZnO [16], ZnS [17, 18], SnO_2_ [19, 20], and (WO_4_) [21] have been widely used in wastewater treatment. Due to its high stability, low cost, nontoxicity, great photoelectric conversion efficiency, and controllable material, ZnO is the most efficient semiconductor photocatalyst. However, ZnO requires UV light for photocatalytic activation [22, 23].

As a result of its wide bandgap energy, narrow visible light absorption, and high recombination rate of photo-generated electron-hole pairs, ZnO only is not applicable [24]. To overcome the limitations of ZnO, different researchers have concentrated on the development of heterojunctions of ZnO with other narrow bandgap semiconductors [25, 26]. There are also reports on doping of metals and nonmetals to improve the catalytic efficiency of ZnO [27–29]. As a result of this modification, the photocatalytic efficiency of ZnO will be improved due the separation of photo-generated electron-hole pairs [30, 31] and improving the visible light absorption of ZnO [32]. Among the materials, Cu-based materials are a promising candidate because they are nontoxic, stable, have a low bandgap, and respond to visible light [33, 34]. Moreover, Cu is suitable for doping as a result of the potential for overlapping the Cu d-electrons with ZnO valance bond [35].

The synthesis of ZnO can be done using a variety of physical and chemical processes [36, 37]. However, the synthesis of materials with plant extract-mediated techniques become promising due to its ecofriendly and simplicity [38–40]. Plant extracts can be used as stabilizing and reducing agents in the synthesis of metal nanoparticles due to the presence of different phenolic groups [41–43]. Such phytochemicals act as the reducing agent to convert the metal salt to the atomic metal state and used as the capping agent to stabilize the particles in the dispersing medium to prevent agglomeration during the synthesis process [44]. On the other hand, the biomediated synthesis method using plant extracts is more advantageous because it does not require hazardous and expensive chemicals and can be processed with low energy [37, 42, 45]. Due to this reason, different reported literature utilized the plant extract-mediated method for enhancing the photocatalytic performance of the catalysts [42, 46]. For instance, Hamad Sadiq et al. synthesized ZnO nanoparticles using *Syzygium cumini* plant leaves extract with a biogenic synthesis approach and used for photocatalytic application [47]. Govindasamy et al. successfully synthesized ZnO nanoparticles through an efficient and facile green synthesis method using *Tecoma castanifolia* leaf extract for enhanced antioxidant activity [48]. Ramin Mohammadi et al. successfully fabricated ZnO and ZnO/CuO nanocomposites using *Mentha longifolia* leaf extract as a natural, nontoxic, and efficient stabilizer [49]. However, there is no report on the synthesis of Cu-doped ZnO using *Eichhornia crassipes* plant extract.

Herein, the Cu-doped ZnO photocatalysts were prepared with the green and coprecipitation approach by using water hyacinth (*Eichhornia crassipes*) aquatic plant extract with varying the amount of copper precursors on a fixed amount of zinc precursors. The resulting catalysts were characterized by using different instruments. The photocatalytic activities of the resulting catalysts were examined on the degradation of methylene blue under visible light irradiation. Furthermore, a possible degradation mechanism with Cu-doped ZnO catalysts was also proposed. Finally, the reusability of the best catalyst was studied systematically. It is expected to attain the higher photocatalytic activities through the synthesis of Cu-doped ZnO photocatalyst materials by using *Eichhornia crassipes* plant extract.

## 2. Materials and Methods

### 2.1. Chemical Regents

Zinc nitrate hexahydrate (Zn (NO_3_)_2_.6H_2_O), copper nitrate trihydrate (Cu (NO_3_)_2_.3H_2_O), sodium hydroxide (NaOH), methylene blue (MB), and ethanol were used in the experiment. All of the chemicals were analytical grade.

### 2.2. Collection and Preparation of Water Hyacinth Extracts

For this experiment, water hyacinth was collected from “Koka Lake,” which is 22.8 kilometers from Adama, Ethiopia. The collected water hyacinth was then washed with distilled water, dried, crushed, and stored at room temperature. Then, crushed water hyacinth powder was boiled for 1 hour at 50°C. Finally, the extract was separated and stored for further application.

### 2.3. Synthesis of Cu-Doped ZnO Photocatalyst

The Cu-doped ZnO photocatalyst *t* was synthesized through a green coprecipitation approach by using water hyacinth extract. In a particular procedure, 0.02445 mole of Zn(NO_3_)_2_.6H_2_O and 0.000247 mole of Cu(NO_3_)_2_.3H_2_0 were added into 100 mL of extract to prepare Cu-ZnO (1%) catalyst. The mixed solution was then stirred for 1 hour using a magnetic stirrer. Then, NaOH was added drop by drop until the pH of the solution reached to 10.35. The precipitate was centrifuged and washed with distilled water and ethanol and then dried in an oven at 80°C for 24 hours. The resulting powder was calcined at 500°C for 2 hours according to the literature report [35]. For all other catalysts, the procedure was similar except varying the amount of copper precursor.

### 2.4. Characterization

The chemical compositions were characterized by X-ray photoelectron spectroscopy (XPS) (ESCALAB 250). The crystal structure of phases of each sample was determined by using the X-ray diffraction instrument (XRD) (XRD-7000S Shimadzu). The field-emission scanning electron microscopy (FE-SEM, JSM 6500F, JEOL) and transmitted electron microscopy (TEM) (FEG TEM technai G2 F30) instruments were used for morphology characterizations. The Shimadzu 3600 Plus UV-vis spectrophotometer was used to check absorption properties of the catalysts and the concentration of the pollutant.

### 2.5. Photocatalytic Performance Evaluation

Photocatalytic experiments were carried out as follows, with a reference to a relevant scientific work [50]. To 125 mL of MB (10 ppm) solution, 25 mg of catalyst was added. The solution was then sonicated for 30 min in the dark to achieve adsorption and desorption equilibrium between the catalyst's surface and the organic dye. Subsequently, the solution was exposed to visible light illumination. Throughout the experiments, the mixture was stirred with a magnetic stirrer. At 20 min intervals, an aliquot was taken and the catalyst was separated from the solution by centrifugation. The degradation of MB dye was analyzed through measuring the change in absorption intensity.

## 3. Result and Discussion

The XRD was used to examine the phase and the crystal structures of the prepared catalysts. As shown in Figure 1, the diffraction peaks for the prepared ZnO, Cu-ZnO (1%), Cu-ZnO (2%), Cu-ZnO (3%), Cu-ZnO (4%), and Cu-ZnO (5%) catalysts were corresponding to the (100), (002), (101), (102), (110), (103), (200), (112), and (201) planes at 2*θ* values of 31.2°, 34.8°, 36.9°, 47.9°, 53.6°, 66.7°, and 75.5°, respectively, in which it is matched with hexagonal wurtzite structure of ZnO (JCPDS No.036-1451). Moreover, a clear additional diffraction peak was observed at 2*θ* of 38.80° on Cu-ZnO/(5%) catalyst. The peak could be related to CuO, which is consistence with literature report [51]. However, in Cu-ZnO (1–4%), the peaks were very small and insignificant as compared to Cu-ZnO/(5%) catalysts due to the smaller amount of CuO in the catalyst, which is also similar with the reported result [52].

The FE-SEM analysis was used to check the surface morphology of the Cu-ZnO (3%) catalyst. Figures 2(a) and 2(b) show the lower and the higher magnification morphologies of the Cu-ZnO (3%) catalyst. As shown in figures, uniformly distributed nearly spherical shaped nanoparticles were observed. Moreover, Figure 2(c) shows the energy dispersive X-ray spectroscopy (EDS) analysis of Cu-ZnO (3%). The EDS clearly shows the existence of Zn, Cu, and O elements in the sample.

The morphological analysis of the Cu-ZnO (3%) catalyst was also further characterized by TEM. As shown in Figures 3(a)–3(c), the lower, medium, and higher-magnification TEM images of the Cu-ZnO (3%) catalyst were indicated, respectively. Furthermore, the HRTEM image of Cu-ZnO (3%) is also shown in Figure 3(d). The effective synthesis of ZnO was confirmed by the lattice fringe with a d-spacing of 0.28 nm in the (002) plane. However, the lattice fringe for CuO was not clearly observed due to the smaller amount of CuO in the sample. Hence, the TEM and HRTEM analysis further confirms the successful preparation of Cu-doped ZnO catalyst.

The chemical composition and oxidation states of the Cu-ZnO (3%) sample were checked by XPS. Figures 4(a)–4(d) show the XPS survey and the spectrum of Zn 2p, Cu 2p, and O 1s peaks, respectively. The peaks from the XPS survey (Figure 4(a)) represented Zn (LMM), Zn 2p_3/2_ and Zn 2p_1/2_, and O 1s. Moreover, Zn 2p_1/2_ and Zn 2p_3/2_ with 1045.38 and 1022.30 eV binding energies, respectively, illustrate the presence of Zn^2+^ in the sample (Figure 4(b)) [53, 54]. As a result, the bonding energy difference between the two peaks was predicted to be around 23.3 eV, which agrees with reported result [55].  Figure 4(c) also indicates the 933.79 and 953.95 eV binding energies, which correspond to Cu 2p_3/2_ and Cu 2p_1/2_, respectively, and attributed to Cu^2+^ [56]. Furthermore, Figure 4(d) shows the O 1s spectra peaks of binding energies at 529.62, 530.58, and 532.1 eV, which indicates the lattice oxygen (ZnO and CuO) and oxygen vacancy, respectively [53, 57, 58].

The optical properties of the pure ZnO and the plant extract mediated Cu-ZnO (3%) catalysts were investigated as shown in Figure 5. As it indicated, ZnO had negligible absorption in the visible light spectral range which is similar with the reported result [59]. However, Cu-ZnO (3%) showed relatively better absorption in the visible light range. The results indicated that the presence of Cu in the ZnO catalyst system could improve absorption in the visible light range which also enhances the photocatalytic activities.

The porosity and specific surface area of Cu-ZnO (3%) was measured by the Brunauer–Emmett–Teller (BET), as shown in the Figure 6. As shown in Figure 6(a), the nitrogen adsorption-desorption isotherms of the Cu-ZnO (3%) catalyst showed the *V* type adsorption-desorption isotherm with a H3 hysteresis loop according to the Brunauer–Deming–Deming–Teller classification [60]. This also confirms the presence of the slit-shaped pore structure according to previous literature [61]. As shown in Figure 6(b), the specific surface area of Cu-ZnO (3%) is 79.9 m^2^/g with pore volume of 0.073 cm^3^/g. Furthermore, the pore size distribution was confirmed to be 1.5687 nm (Figure 6(b)). Therefore, this result indicates that enhanced specific surface area of Cu-ZnO (3%) is achieved through using water hyacinth extract as a template which is better as compared to previous literature [49].

The photocatalytic performances of the prepared catalysts were examined on degradation of MB dye.  Figure 7(a) shows the UV-vis absorption spectra for the Cu-ZnO (3%) catalyst at different irradiation times under visible light. As shown in Figure, the concentration of MB dye was changed as the photocatalytic reactions proceed. Moreover, the *C*_*t*_/*C*_*0*_ ratio, where *C*_*0*_ is the initial concentration and *C*_*t*_ is the concentration of MB after time (*t*) in min, was calculated and is shown in Figure 7(b). As shown in Figure 7, Cu-ZnO (3%) showed the best photocatalytic performance and degrades 89% of the MB dye. However, the degradation performances of blank (without catalysts), ZnO, Cu-ZnO (1%), Cu-ZnO (2%), Cu-ZnO (4%), and Cu-ZnO (5%) catalysts were 6, 54, 69, 83, 80, and 73%, respectively.

According to the Langmuir–Hinshelwood (L–H) model [62], the rate expression is given by

(1) $$\begin{array}{c} \ln\left(\frac{C_{t}}{C_{0}}\right)=-kt, \end{array}$$

where *C*_*t*_ is the concentration at time *t*, *C*_*0*_ is the initial concentration of the dye, and *k* is the apparent first-order rate constant [14].  Figure 7(c) shows a plot of ln *C*_*t*_/*C*_*0*_ versus time. Because of the linear relationship between ln (*C*_*t*_/*C*_*0*_) and their respective irradiation time, the photocatalytic degradation reaction for this experiment was proven to follow pseudo-first-order kinetics [63]. The rate constants of ZnO, Cu-ZnO (1%), Cu-ZnO (2%), Cu-ZnO (3%), Cu-ZnO (4%), and Cu-ZnO (5%) catalysts were calculated and indicated as 0.0063, 0.00972, 0.0159, 0.0195, 0.0126, and 0.01099 min^−1^, respectively.

The degradation mechanism of MB dye with Cu-ZnO (3%) catalyst is shown in Figure 8. It is known that the photocatalyst can absorb light to generate electron and hole pairs. After exposing to light irradiation, the electrons excitation into the conduction band (CB) occurred. Simultaneously, the holes remained in VB of semiconductors [64]. After doping of Cu into ZnO, the electrons and holes recombination will be suppressed by trapping of electrons [23, 28]. Then, the electrons remained on the surface of the catalyst and interacted with the adsorbed O_2_ to generate a superoxide radical anion (O_2_). The holes can also react with H_2_O, and hydroxyl radical (OH) will be formed. The reactive oxygen species (ROS) are responsible in the degradation of organic dye [65–67]. Figure 8 shows the possible degradation mechanism of MB dye.

## 4. Conclusion

The green method using unwanted water hyacinth plant extract in the preparation of Cu-ZnO photocatalysts is reported. The amount of copper content was also optimized, and Cu-ZnO prepared with 3% of molar ratio of the copper precursor showed a good catalytic activity. Cu-ZnO (3%) degrades 89% of the MB dye, while the degradation performances of blank (without catalysts), ZnO, Cu-ZnO (1%), Cu-ZnO (2%), Cu-ZnO (4%), and Cu-ZnO (5%) catalysts were 6, 54, 69, 83, 80, and 73%, respectively. The presence of water hyacinth plant extract in the preparation of Cu-ZnO enhances the porosity and visible light absorption. As a result, the photocatalytic activity of ZnO could be enhanced. Moreover, the impurity level resulted from Cu-doping promote the synergetic effect through suppressing the charge carriers recombination rate and shifting the conduction band to lower energy level for overall enhancement of photocatalytic degradation of methylene blue.

## Figures and Tables

**Figure 1:** XRD diffraction patterns of (a) ZnO, (b) Cu-ZnO (1%), (c) Cu-ZnO (2%), (d) Cu-ZnO (3%), (e) Cu-ZnO (4%), and (f) Cu-ZnO (5%).

**Figure 2:** (a-b) SEM image of lower and higher magnifications, and (c) the EDS analysis for Cu-ZnO (3%) with plant extract.

**Figure 3:** (a–c) TEM image of lower, medium, and higher magnification and (d) HRTEM images of Cu-ZnO (3%) catalyst with plant extract.

**Figure 4:** (a) XPS survey and spectra of (b) Zn 2p, (c) Cu 2p, and (d) O 1s for Cu-ZnO (3%) with plant extract.

**Figure 5:** The UV-visible spectra of the ZnO and Cu-ZnO (3%) catalysts.

**Figure 6:** (a) Nitrogen adsorption-desorption isotherms and (b) pore size distribution curves for Cu-ZnO (3%) with plant extract.

**Figure 7:** (a) UV-vis absorption spectra of Cu-ZnO (3%) and (b) *C*_*t*_/*C*_*0*_ plots and (c) the first-order kinetic plot for ZnO, Cu-ZnO (1%), Cu-ZnO (2%), Cu-ZnO (4%), and Cu-ZnO (5%) catalysts.

**Figure 8:** The possible degradation mechanism of MB dye with Cu-ZnO photocatalyst.

## Data Availability

The data used to support the findings of this study are included within the article.
